# Nontuberculous Mycobacterial Resistance to Antibiotics and Disinfectants: Challenges Still Ahead

**DOI:** 10.1155/2022/8168750

**Published:** 2022-02-26

**Authors:** Samira Tarashi, Seyed Davar Siadat, Abolfazl Fateh

**Affiliations:** ^1^Department of Mycobacteriology and Pulmonary Research, Pasteur Institute of Iran, Tehran, Iran; ^2^Microbiology Research Center (MRC), Pasteur Institute of Iran, Tehran, Iran

## Abstract

The mortality incidence from nontuberculous mycobacteria (NTM) infections has been steadily developing globally. These bacterial agents were once thought to be innocent environmental saprophytic that are only dangerous to patients with defective lungs or the immunosuppressed. Nevertheless, the emergence of highly resistant NTM to different antibiotics and disinfectants increased the importance of these agents in the health system. Currently, NTM frequently infect seemingly immunocompetent individuals at rising rates. This is of concern as the resistant NTM are difficult to control and treat. The details behind this NTM development are only beginning to be clarified. The current study will provide an overview of the most important NTM resistance mechanisms to not only antibiotics but also the most commonly used disinfectants. Such evaluations can open new doors to improving control strategies and reducing the risk of NTM infection. Moreover, further studies are crucial to uncover this association.

## 1. Introduction

Accumulated evidence confirmed the global importance of nontuberculous mycobacteria (NTM) as one of the alarming sources of opportunistic infections in human history [1]. The NTM refer to mycobacteria species other than the *Mycobacterium tuberculosis* complex and *M. leprae* [2]. More than 200 NTM species were identified and some of which are known as important infectious threats, especially in industrialized countries [3, 4]. These bacterial agents exist ubiquitous in the environment and are ubiquitously transmitted by inhalation, ingestion, or direct inoculation in the skin to develop infections [5]. Different NTM species are distinct based on their growth rate, rapid (*e.g*., *M. abscessus*, *M. chelonae*, and *M. fortuitum*) and slow growers (*e.g*., *M. avium complex* and *M. kansasii*). Additionally, *M. marinum* was introduced as an intermediate category between rapid and slow growers [6, 7].

The variety between different NTM species faces clinical laboratories with high challenges in the accurate detection of a real infectious agent, and following it makes high complexity in the detection of exact antibiotic susceptibility, drug regimens, and treatment outcomes [8, 9]. In light of the wide variety of NTM species and their importance in clinics, effective control and proper drug prescription are crucial [10].

Drug susceptibility testing (DST), as an established tool in a laboratory, traditionally plays a significant role in the delineation of the most effective drug regimens in different NTM infections [11, 12]. Nevertheless, there are important discrepancies between the results of DST measured *in vitro* and the effectiveness of selected drugs *in vivo* for several drugs except for macrolides and amikacin [13]. These shortcomings are partly driven by a lack of standardized laboratory methods, efficient control strategies, and monitoring. However, it should be noted which NTM infections are increasingly detected in clinics; therefore, giving attention to DST should not be neglected [14]. To date, limited studies have focused on acquired resistance mechanisms associated with NTM infections against antibiotics and disinfectants [15, 16]. The current study provides a summarized overview of the mechanisms of drug resistance and drug regimens in NTM infections. The importance of disinfectants and detection of NTM species is briefly conferred as the scope of this review.

## 2. Importance of Antimicrobial Resistance Mechanisms of NTM Species

The effective treatment of NTM infections is highly challenging owing to several factors, such as costliness, time-consumingness, toxicities, poor outcome, and appearance of resistance at high levels. Resistance might be either intrinsic or acquired. The NTM are intrinsically resistant by some mechanisms, such as impermeable cell walls, thickness, and formation of granulomas which effectively decrease antimicrobial influx and protein expression that target antibiotics. On the other hand, acquired resistance is generally related to prolonged antibiotic prescription required to treat NTM infections.  Figure 1 illustrates the most probable intrinsic and acquired resistance mechanisms detected in NTM species. The utility of *in vitro* DST for handling NTM infections remains challenging due to incompatibility between DST results and clinical outcomes [8, 17]. Nevertheless, a standardized DST still plays a significant role in the choice of the most effective drugs for the most optimized treatment of different NTM infections, particularly for rapid growers.

For the most effective control, the Infectious Diseases Society of America (IDSA) and the American Thoracic Society (ATS) introduced some valuable diagnostic criteria for the evaluation of patients suspected of NTM pulmonary infections and prescription of appropriate drug regimens [17]. In addition, the Clinical and Laboratory Standards Institute (CLSI) addressed some criteria and recommendations for DST based on organism distribution, clinical data, and the experience of NTM infections [7]. A clear association has been detected for some drugs and special NTM infections [8, 18]. Different drugs have been affecting the targeted sites by several mechanisms such as suppression of cell wall synthesis, suppression of DNA synthesis, suppression of protein synthesis, and suppression of respiratory chain (Table 1).

Usually, the recommended drug regimen for most slow growers consists of ethambutol, rifampicin, and a macrolide. If the related infection is severe, amikacin or streptomycin can be added. In the case of rapid growing infections, the drug therapy is primarily prescribed based on the *in vitro* results of DST. In these cases, DST is typically performed for macrolides, aminoglycosides, fluoroquinolones, amikacin, imipenem, tetracyclines, linezolid, and trimethoprim-sulfamethoxazole [17]. The rate of successful treatment of NTM infections is related to the species type (e.g., 30-50% in *M. abscessus*, 50-70% in *M. avium* complex, and 80-90% in *M. malmoense* and *M. kansasii* infections) [19]. Based on the results of the IDSA, ATS, and CLSI, the most important resistant mechanisms identified for previously proper NTM drug regimens consist of macrolides, quinolones, clofazimine, linezolid, bedaquiline, aminoglycosides, sulfonamides, and tetracyclines [20].

Conceptually, the development and employment of novel, safe, and more effective drugs count as a crucial medical need to treat NTM infections. Although numerous evaluations have focused on different aspects of NTM isolates, there have still been many questions in this research area. The subsequent sections will discuss the informed data on the action and resistance mechanisms of each effective evaluated drug in NTM infections.

### 2.1. Suppression of Cell Wall Synthesis

#### 2.1.1. Ethambutol

Ethambutol is one of the major agents in drug regimens of patients with some NTM slow growers, such as *Mycobacterium avium* complex (MAC) and *M. kansasii* infections. The prescription of this agent is limited for rapid growers of NTM infections [20]. Ethambutol disrupts the cell wall by the suppression of biosynthesis of arabinogalactan and, to a lesser extent, lipoarabinomannan [21]. Ethambutol resistance is acquired by a mutation in the *embCAB* gene, frequently in codon 306 of the *embB* gene, which leads to the inhibition of mycobacterial arabinosyl transferase translation [22]. *M. kansasii* acquired ethambutol resistance by M306I substitution in *embB*, in addition to G406P and M423I alterations [23]. *M. avium* acquired ethambutol resistance by the overexpression of *embAB* genes. *M. smegmatis* acquired this resistance by a point mutation in the *embB* gene. However, the main genetic diversity for the ethambutol resistance of *M. kansasii* and MAC is still unidentified. The intrinsic mechanism of ethambutol resistance is still uncharacterized, although *embB* polymorphisms might be associated with its intrinsic resistance in some NTM species [24].

#### 2.1.2. Beta-Lactams

Beta-lactams are prescribed as antituberculosis agents, and clinically acquired resistance to them has not been reported for NTM species [20]. Furthermore, their intrinsic resistance might appear due to the effects of cell wall permeability, the affinity of penicillin-binding proteins (PBP), and the activity of *β*-lactamases [25]. Several studies indicated the effects of each mechanism on NTM species. For example, the effect of cell wall permeability was previously evaluated in *M. fortuitum*, *M. chelonae*, and *M. smegmatis* [25–27]. The association between the affinity of PBP and *β*-lactams resistance of some NTM species was also assessed in *M. fortuitum*, *M. smegmatis*, and *M. abscessus* [27, 28]. Finally, the effect of *β*-lactamases was reported in the resistance of *M. avium*, *M. abscessus*, *M. fortuitum*, and *M. smegmatis* to different agents of *β*-lactams [29]. The only recommended beta-lactam for mycobacterial infections is imipenem that is specifically used for rapid growers of NTM such as *M. chelonae*, *M abscessus*, and *M. fortuitum* [30, 31].

#### 2.1.3. Isoniazid

Isoniazid showed potent activity against some NTM species, such as *M. kansasii* and *M. xenopi* [32]. The action of this agent is based on the inhibition of mycolic acid synthesis by targeting the acyl carrier protein (ACP) reductase, the fatty acid synthesis II (FAS II) enzymes, the FAS II enzyme *β*-ketoacyl-AcpM synthase (KasA), InhA, or dihydrofolate reductase (DHFR). Overall, most species of NTM are intrinsically resistant to isoniazid due to the lack of catalase-peroxidase KatG, which is necessary for its action [20]. The presence of an isoniazid efflux pump may also lead to its resistance [33]. The acquired resistance of isoniazid to NTM was not comprehensively evaluated [20].

#### 2.1.4. Vancomycin

Vancomycin is commonly used in clinics against some NTM infections; however, most NTM infections are intrinsically resistant to this agent [20]. Vancomycin inhibits mature peptidoglycan assembly. The reason for the highest NTM resistance to vancomycin is the presence of canonical binding sites for vancomycin in the mycobacterial peptidoglycan, which might enhance cell wall permeability [34]. The best-known mechanism for acquired resistance to vancomycin is generally the presence of VanA or VanB; nevertheless, it has not been defined for NTM species [20].

#### 2.1.5. Delamanid

Delamanid is derived from nitro-dihydro-imidazooxazole and often used in drug regimen of patients infected with multidrug-resistant tuberculosis [35]. This agent is also a potential choice of drug regimen of *M. intracellulare* and *M. avium* infection [36]. Delamanid inhibits synthesis of keto- and methoxy-mycolic acid [35]. Its resistance among *M. tuberculosis* strains is infrequent. Nevertheless, increasing evidence highlighted its resistance tendency and prolonged treatment courses. The resistance mechanism to delamanid has not been well identified for NTM isolates [10]. It is reported that MIC value of delamanid is very variable and higher resistance has been showed for *M. kansasii* [37, 38].

### 2.2. Suppression of DNA Synthesis

#### 2.2.1. Fluoroquinolones

Fluoroquinolones are often suggested for macrolide-resistant MAC and *M. abscessus* [8, 18]. Their action is dependent to inhibition of DNA synthesis by disruption of topoisomerase IV and DNA gyrase, two involved key enzymes in DNA supercoiling [31]. Resistance mechanism to fluoroquinolones is usually introduced by disruption in DNA gyrase through mutations in the quinolone resistance-determining region (QRDR) of *gyrA* and *gyrB* genes [39]. Nevertheless, the frequency of *gyrA* and *gyrB* mutations in MAC was reported in only a few studies, and conflicting results were conveyed for *M*. *abscessus* isolates [40, 41]. In other words, several studies showed fluoroquinolone resistance without any reports of *gyrA* and *gyrB* mutations in NTM infections [23, 40]. Therefore, further investigations are required to confirm the responsible loci for fluoroquinolone resistance in addition to the QRDR of *gyrA* and *gyrB*. Along with the *gyrA* and *gyrB*, topoisomerase IV is also a target of fluoroquinolones. Topoisomerase IV was not encoded in pathogenic NTM, such as *M. avium* and *M. abscessus*; however, *M. smegmatis* and *M. vanbaalenii* encode this enzyme [20]. In addition, the LfrA efflux pump was introduced in NTM resistance; nonetheless, the importance of this mechanism is unclear [42].

#### 2.2.2. Trimethoprim and Sulfonamides

Sulfamethoxazole, as an important agent of trimethoprim and sulfonamides, inhibits microbial folate metabolism and reduces nucleic acid synthesis [43]. Their resistance has been indicated in NTM infections; however, underlying mechanisms have not been often explained. The intrinsic trimethoprim resistance in *M. avium* and *M. smegmatis* correlates with dihydrofolate resistance of reductase [44].

#### 2.2.3. SPR719 and SPR720

Recently, SPR719 and SPR720 (prodrug of SPR719) were introduced as a novel aminobenzimidazole by the inhibition of the ATPase activity gyrase and topoisomerase IV [16, 45]. Preliminary analysis has confirmed the antimicrobial efficacy of SPR719/720 against sensitive and multiple-drug resistant *M. tuberculosis* [46]. In addition, its positive effect on MAC, *M. abscessus*, and *M. kansasii* has been detected [46, 47]. Further advancement of this novel agent is required for the most efficient treatment of NTM infections.

### 2.3. Suppression of Protein Synthesis

#### 2.3.1. Macrolides

Clarithromycin and azithromycin, as two types of macrolides, are known as key drugs for NTM therapy among most physicians [8, 18]. They show the elongation of peptide chains by binding to the peptide that is the exit tunnel of the ribosome. Resistance mechanisms to clarithromycin and azithromycin are almost always acquired by a specific mutation, nucleotides 2058 and 2059, in the *23S rRNA* gene, which was identified in the early 1990s [15]. These mutations caused a base alteration in the critical rRNA position (A2058 or A2059) involved in binding macrolides and ribosomes. These point mutations have been identified in clinical macrolide-resistance MAC isolates at high frequencies [48]. Moreover, the acquisition of these point mutations was identified in *M. abscessus*, *M. fortuitum*, *M. kansasii*, and *M. chelonae* [49]. In addition, resistance might be induced by encoding a ribosomal methyltransferase by the *erm* genes, including *erm*(38), *erm*(39), *erm*(40), and *erm*(41) [20]. This resistance mechanism is identified in *M. abscessus*, *M. goodie*, *M. smegmatis*, *M. boenickei*, *M. houstonense*, *M. neworleansense*, *M. fortuitum*, *M. porcinum*, *M. mageritense*, *M. wolinskyi*, and *M. bolletii* infections [50, 51]. The inducible macrolide resistance does not occur in *M. massiliense* due to the deletion of the *erm*(41) gene [52]. Therefore, *M. massiliense* has a better response to macrolide-based treatments [53]. *M. abscessus* and *M. massiliense* might also acquire macrolide resistance by a point mutation in the *23S rRNA* gene [54].

#### 2.3.2. Oxazolidinones

Linezolid and tedizolid are both used against NTM infections. Linezolid is often recommended for the therapy of MAC and *M. abscessus* [55]. This agent binds the 23SrRNA and suppresses protein synthesis. The resistance mechanism of linezolid, described in *M. tuberculosis*, is acquired by a mutation in *rplC* and *23S rRNA* genes, which is distinct from mutations involved in macrolide resistance [56]. These mutations cause the inhibition of protein synthesis by binding to the peptidyl ribosomal transferase. The appearance of extensive toxicity after the prolonged use of linezolid was identified as a significant concern in clinical practice. Therefore, tedizolid and LCB01-0371 are recently developed as more acceptable alternative agents to linezolid [57]. LCB01-0371, as a novel oxazolidinone in phase II clinical experiments, showed potential activity against *M. abscessus* infections [58]. However, the resistance mechanism, efficacy, and tolerability of linezolid and tedizolid have not yet been defined for NTM isolates [10].

#### 2.3.3. Aminoglycosides

Amikacin, gentamicin, kanamycin, and tobramycin are known as major members of aminoglycosides. Recently, the administration of liposomal amikacin for inhalation was introduced as a high-effectiveness agent against the majority of NTM species [15, 59]. These agents disturb the translation process and cause cell death by irreversibly binding to the 30S ribosomal subunit of bacteria. Resistance mechanism to them might be primarily acquired by a unique mutation in the *16S rRNA* gene (*rpsL*) gene that leads to the modification of the 30S ribosomal subunit [20]. This point mutation, A1408G, is detected in MAC, *M. chelonae*, *M. massiliense*, and *M. abscessus* [41, 60]. Additional mutations, T1406A, C1409T, and G1491T, associated with aminoglycoside resistance were also observed in *M. abscessus* [61]. Acetyltransferase inactivates aminoglycosides and plays a significant role in acquired and intrinsic resistance to these agents in NTM infections similar to other bacteria [20]. In addition, aminoglycoside phosphotransferases are expressed by some resistant NTM species, including *M. fortuitum*, *M. abscessus*, and *M. avium* [62]. Nevertheless, some evaluations indicated that resistance by aminoglycoside phosphotransferases is likely to be unusual for most NTM species [20].

#### 2.3.4. Tetracyclines

Tetracycline and doxycycline reversibly bind to the 30S ribosomal subunit at multiple points and suppress protein synthesis [63]. They block binding of tRNA and mRNA-ribosome complex and inhibit elongation of peptides. Tetracycline resistance NTM is acquired by ribosome protection proteins expressed by *otr*(A) and *tet*(M) genes, which are homologous critical elongation factors for correct ribosome function [64]. In addition, the increased resistance of tetracyclines in NTM species is acquired by Tet and Otr efflux pumps, which is homologous with some founded genes in other bacteria, such as *tet*(L), *tet*(K), *tet*(V), and *otr*(B). Tap was introduced as a specific tetracycline efflux pump NTM species [65].

#### 2.3.5. Tigecycline

Tigecycline was recently introduced as potential agents against NTM infections. Tigecycline is typically prescribed in *M. abscessus* infections; however, its use is limited due to probable side effects [66]. Overall, tigecycline has been introduced as the only practical drug in the chemotherapy of *M. abscessus* and *M. chelonae* infections [66]. This agent suppresses protein synthesis by binding to 30S ribosomal subunit and preventing the acyltRNA binding. However, tigecycline resistance might be acquired by Tet(X) enzyme; nevertheless, its common acquired resistant mechanisms have not yet been conferred for clinical NTM species [67].

#### 2.3.6. Rifampin

Similar to ethambutol, rifampin is one of the key agents for the drug regimens of patients with *M. kansasii* and MAC infections. This agent suppresses the DNA-dependent RNA polymerase of bacteria by binding to it that is encoded by the *rpoB* gene. Rifampin resistance is acquired by a mutation in a unique region of the *rpoB* gene that is identified as the rifampicin-resistance-determining region (RRDR) [68]. The *rpoB* gene encodes the *β*-subunit of bacterial RNA polymerase [15]. The mutation in the RRDR is often detected in *M. kansasii* than MAC. Several clinical isolates of MAC and *M. ulcerans* were identified by harbored mutations in the *rpoB* gene (including codons 513, 516, 526, and 531 of RpoB) [69]. *M. smegmatis* and *M. abscessus* intrinsically reduced the function of rifampin by the expression of the *arr* gene [20]. Overall, resistance to rifampin and clarithromycin should be tested in induced infections by *M. kansasii* and MAC isolates [11].

### 2.4. Suppression of Respiratory Chain

#### 2.4.1. Bedaquiline

Bedaquiline is mostly suggested in drug regimens of multidrug-resistant tuberculosis and *M. leprae*. Bedaquiline has been recently prescribed for MAC and *M. abscessus* infections [70]. A study exhibited the highest activity of bedaquiline against *M. avium*, *M. abscessus*, and *M. massiliense* than *M. fortuitum* [71]. Bedaquiline action is dependent to suppression of NTM respiratory chain. This agent suppresses the product of the *atpE* gene, a mycobacterial ATP synthase, and leads to cell death because of lack of ATP production [72, 73]. Resistance mechanisms to bedaquiline are acquired by mutations in *atpE*, *mmpT5*, and *pepQ* genes [71, 74]. Some NTM isolates, such as *M. avium*, *M. intracellulare*, *M. kansasii*, *M. abscessus*, *M. flavescens*, *M. massiliense*, and *M. fortuitum* isolates, have infrequently shown mutations in *atpE* [71, 75]. Some bedaquiline resistance *M. intracellulare* isolates also showed mutations in *mmpT5* [74]. A cross-resistance has been strongly exhibited between bedaquiline and clofazimine in *M. tuberculosis* [76]. Overall, further evaluations are required for a better understanding of bedaquiline resistance mechanisms in NTM infections.

#### 2.4.2. Clofazimine

Clofazimine has been prescribed in drug regimens for MAC and *M. abscessus* infections since the 1990s [77]. The oral administration of clofazimine is well tolerated in almost all species of NTM [78]. Moreover, the real action of clofazimine is not well described; nevertheless, available evidence has suggested that it inhibits bacterial proliferation by binding to its DNA strand and blocking the function of template strands of DNA and intracellular redox cycling [77]. In addition, this drug agent might interrupt bacterial cell membranes by affecting phospholipids. Resistance mechanism to clofazimine is frequently identified in *M. tuberculosis* by mutations in the *mmpR5* and occasionally in the *pepQ* genes [79]. The *mmpL5* mutations lead to the limitation of encoding a transcriptional regulator by *mmpL5*, thereby inducing the expression of an efflux pump, MmpS5-MmpL5 [79]. Some mutations related to clofazimine resistance were also identified in *M. abscessus*, such as MAB_0540, MAB_2299c, and MAB_1483 [80]. *M. intracellulare* also showed some mutations in the *mmpL5* gene. However, *M. avium* isolates, despite being clofazimine-resistant, did not show any related mutations [81]. Such results highlighted the need for further evaluation of clofazimine resistance in NTM infections.

## 3. Importance of Disinfection Mechanisms of NTM Species

As previously mentioned, NTM isolates commonly exist ubiquitously and are easily transmitted, particularly among hospital patients. It is assumed that the source of the majority of NTM infections is environmental NTM [82]. Considering that there is no optimized detection and treatment against NTM isolates, appropriate strategies need to be taken to minimize and control their spread [83]. Therefore, sterilization and use of disinfectants play a crucial role in proper NTM control, especially in medical care units [84]. Nonetheless, different NTM species have presented strong resistance to different disinfectants and have typically drawn more attention in the studies related to disinfectant-resistant bacteria [85]. The most important reasons for disinfectant-resistant NTM are their thick, waxy, and hydrophobic cell surface rich in mycolic acids, clump formation, and accumulation in the biofilms [86]. It is required to introduce an economical and effective disinfectant against NTM species. The subsequent sections will discuss the effect of some disinfectants on NTM species.

### 3.1. Chlorine and Ozone

The NTM species are more resistant to chlorine and ozone disinfection. Their activity is dependent on the strain, concentration, time of interaction with NTM species, and other environmental factors, such as pH, temperature, and condition of isolation of NTM species (isolated from culture media or natural water) [86]. As a strong sterilization system with a low cost, chlorination is often used to obtain high-quality water and offers residual disinfection [82, 83]. However, some bacteria, particularly several NTM isolates, can overwhelm chlorine disinfection [84, 87]. Some studies reported the high viability of *M. fortuitum* and *M. avium* rather than *Escherichia coli* during chlorine disinfection [87, 88]. In addition, high tolerance of *M. chelonae*, *M. mucogenicum*, *M. fortuitum*, *M. gordonae*, and *M. aurum* against chlorine disinfection has been reported [87, 89]. To date, despite the high importance of NTM isolates during chlorine disinfection, the influencing mechanisms and factors have rarely been evaluated. The formation of being spiked with *M. terrae* increases the aggregation and clump formation of NTM, specifically in wastewater, and is a strong reason for the chlorine resistance of *M. terrae* [5].

### 3.2. Glutaraldehyde and Amine

Glutaraldehyde-resistant strains of *M. chelonae* and peracetic acid-resistant strains have been isolated from environmental samples. It is vague whether the glutaraldehyde resistance of *M. chelonae* is an acquired or intrinsic characteristic. Even a mixture of several aldehydes cannot overcome glutaraldehyde-resistant strains. Therefore, an alternative disinfectant, such as glucoprotamin, might show beneficial effects. Glucoprotamin is introduced as a new amine derived that often shows good efficiency against most of the different NTM isolates, such as *M. smegmatis*, *M. avium*, *M. kansasii*, *M. terrae*, and *M. xenopi*, except for *M. chelonae* [90, 91]. Most other disinfectants are not notably efficient in *M. avium*. *M. bolletii* and *M. massiliense* have indicated more resistance against an acetic acid solution [92].

### 3.3. Ultraviolet Irradiation

Ultraviolet (UV) radiation has been revealed as the most effective sterilization system in the inactivation of most microbes by affecting DNA. However, limited evidence showed the mechanism of UV radiation's impact on the inactivation of NTM species [86]. The NTM species are likely more resistant to sterilization methods by UV radiation. Two studies previously reported the UV inactivation of *M. tuberculosis* and *M. avium* based on dosimetry [93]. Nevertheless, the detailed dosimetry of these studies was not confirmable according to the details of the publications. In addition, the resistance of *M. terrae* to UV radiation was observed because it tended to aggregation and clump formation [86]. Other studies reported that the complete elimination of *M. fortuitum* needed a longer time or dose of UV exposure rather than *M. marinum* [83, 94]. Moreover, the impact of UV radiation on the inactivation of *M. avium* and *M. intracellulare* is measured [95].

### 3.4. Other Disinfectants

The efficacy of calcium hypochlorite against *M. fortuitum* was reported higher than that against *M. marinum* [83]. A study introduced some available agents for efficacy against NTM infections and general disinfection of equipment in the aquaculture industry [96]. For example, it is stated which sodium hypochlorite at high doses is required for NTM infections. Additionally, formaldehyde is known as a highly effective agent against NTM species; nonetheless, it is a potential carcinogen and is usually used for equipment. Alcohols are commonly used for equipment and surfaces; however, the resistance of some NTM to these compounds has been reported [97]. In addition, quaternary ammonia, iodophors, phenolics, and autoclave tools can be effective against NTM species. The results of another study indicated higher resistance of *M. immunogenum* than other tested organisms against formaldehyde, isothiazolone, and phenolic biocide [98].

## 4. Summarized Points in DST of NTM Species

With regard to the variability of NTM species in the results of drug therapy and outcomes, their accurate identification and standard antibiotic susceptibility attracted great interest [99]. The first consensus document on the DST of mycobacteria was published in 1963 [100]. For several years, different methods for DST of NTM isolates have been tested [13, 20]. The common techniques for DST in bacteriology laboratories are typically used for rapid growers of NTM species; nevertheless, unique DST methods designed for *M. tuberculosis* are often applied to slow growers. The foundation of different methods of DST is based on three procedures, including the absolute concentration, resistance ratio, and proportion methods [13]. The cutoff point of resistance is provided for all three methods. This was derived based on the determination of the minimum inhibitory concentration (MIC) of series wild-type *M. tuberculosis* which is isolated from patients who had no contact with other patients under antituberculosis treatment [100]. Among these three procedures, the resistance ratio method is frequently used for *M. tuberculosis* than NTM isolates [101].

The determination of MICs is often based on absolute concentration methods. The MICs are broadly adapted for DST NTM isolates; nevertheless, MIC resistance cutoff points have not been correctly determined and clinically validated [102]. The determination of MIC is according to inoculating broth media and various concentrations of drugs to be tested for critical concentration of inhibitory of standardized inoculated NTM isolates. The resistance is defined as growth over than 1 : 100 dilution of inoculum of medium without the drug [100]. Generally, MICs are based on broth macrodilution or broth microdilution. Two main methods for broth macrodilution include BacTec 460 and Mycobacterial Growth Indicator Tube (MGIT) [13]. The broth macrodilution is usually defined for slow growers, and due to difficulty in clinical results in their interpretation, these methods are less approved for rapid growers of NTM [13]. However, the suitability of broth microdilution is confirmed for rapid growers of NTM species. Furthermore, this method is developed for slow growers by applying the Middlebrook 7H9 medium [103].

The disk diffusion method is based on the proportion method. The foundation of this method is placing a disk with the standard quality of a unique drug on an agar medium which is inoculated by the test isolate [7]. The results are interpreted based on the inhibition zone of growth. The utility of this method is difficult to adapt for slow growers of NTM. Therefore, to provide the growth of all NTM species, some booster factors, such as albumin, catalase, oleic acid, and dextrose, were added to the agar medium [104]. In addition, disk elution was approved for the DST of some NTM isolates, such as *M. fortuitum* and *M. marinum* [105]. In this method, the fixed quantities of drugs are added to the medium, and the results are determined based on growth or no growth at a related concentration [7].

Epsilon tests are termed “E-tests,” known as a strip standardized with a continuous logarithmic MIC measurement that covers 15 twofold dilutions of the test drug. The related strips are placed on an agar medium in which a suspension of NTM isolates with a preset inoculum is swabbed [13]. The most significant limitation of E-tests' utility for NTM isolates, particularly for rapid growers, is that they were calibrated for MIC readings after 18-24 hours of incubation [13].

Most resistant NTM isolates harbor unique mutations, which are pointed in the previous sections, easily detected by different molecular methods [13]. The utility of sequencing some target genes and comparisons with related reference genes of wild-type strains of the same species have been developed, particularly for MAC, *M. abscessus*, and *M. kansasii* [13, 50, 60]. Such methods count as beneficial tools to confirm the relationship between particular susceptibility profiles and clinical impact [13]. With time, introducing the whole genome sequencing method suppressed earlier molecular tests, such as single-target sequencing methods and line probe assays [13].

## 5. Perspectives

Emerging scientific evidence on the importance of resistance in NTM infections continues to be clarified and refined. Currently, due to the widespread use of disinfectants, particularly on account of the marked coronavirus disease 2019 pandemic, resistance to disinfectants needs to be better clarified than antibiotics in this field. Generally, the evaluations of NTM resistance can be typically effective in devising innovative control strategies and fighting for their development; therefore, such evaluations have become an urgent topic for future research. This study tried to provide an overview of the resistance mechanisms of the salient antibiotics and disinfectants during different NTM infections.

## Figures and Tables

**Figure 1:** The most probable resistance mechanisms in NTM infections.

**Table 1:** Characteristics of used antibiotics in NTM infections based on action and resistance mechanisms.

	Antibiotic	Action mechanism	Resistance mechanism	Highest activity against	Lowest activity against
Suppression of cell wall synthesis	Ethambutol	Suppression of arabinogalactan biosynthesis	Mutation in *embCAB* and inhibition of mycobacterial arabinosyl transferase translation	Rapid growers of NTM MAC^1^ *M. kansasii*	*M. kansasii* *M. avium* *M. smegmatis*
	Beta-lactams (imipenem)	Suppression of enzymatic activity of PBPs^2^ and peptidoglycan synthesis	Enhance cell wall permeability, the affinity of PBP, and the activity of *β*-lactamases	Rapid growers of NTM	*M. fortuitum* *M. chelonae* *M. smegmatis* *M. abscessus* *M. avium*
	Isoniazid	Suppression of mycolic acid synthesis	Lack of catalase-peroxidase KatG and isoniazid efflux pump	*M. kansasii* *M. xenopi*	Most species of NTM
	Vancomycin	Suppression of mature peptidoglycan assembly	Enhance cell wall permeability	Most species of NTM	Most species of NTM
	Delamanid	Suppression of keto- and methoxy-mycolic acid synthesis	Not determined for NTM species	MDR-TB^3^ M*. intracellulare* *M. avium*	*M. kansasii*

Suppression of DNA synthesis	Fluoroquinolones	Suppression of topoisomerase IV and DNA gyrase	Mutations in *gyrA* and *gyrB* genes LfrA efflux pump The main mechanism is not clear	Macrolide-resistant MAC *M. abscessus*	MAC *M*. *abscessus* *M. smegmatis* *M. vanbaalenii*
	Sulfamethoxazole	Suppression of microbial folate metabolism and nucleic acid synthesis	Activity of reductase	Most species of NTM	*M. avium* *M. smegmatis*
	SPR719 and SPR720	Suppression of ATPase activity gyrase and topoisomerase IV	Not determined for NTM species	*M. tuberculosis* MAC *M. abscessus* *M. kansasii*	Not determined for NTM species

Suppression of protein synthesis	Macrolides (clarithromycin and azithromycin)	Suppression of peptide chain elongation by binding to the exited peptide from ribosome	Activity of ribosomal methyltransferase (erm) Mutation in *23SrRNA*	Most species of NTM	*M. bolletii* *M. goodie* *M. kansasii* *M. chelonae* *M. abscessus* *M. wolinskyi* *M. boenickei* *M. fortuitum* *M. porcinum* *M. smegmatis* *M. massiliense* *M. houstonense* *M. mageritense* *M. neworleansense*
	Oxazolidinones (linezolid, tedizolid, and LCB01-0371)	Binding to the 23SrRNA and suppression of protein synthesis	Mutation in *rplC* and *23SrRNA*	Most species of NTM (linezolid for MAC and *M. abscessus*)	*M. tuberculosis* Not determined for NTM species
	Aminoglycosides	Irreversible binding to the 30S ribosomal subunit and suppression of translation process	Mutation in *16SrRNA* (*rpsL*) Activity of phosphotransferases and acetyltransferase	Most species of NTM	MAC *M. chelonae* *M. massiliense* *M. abscessus* *M. fortuitum* *M. avium*
	Tetracyclines	Reversibly bind to the 30S ribosomal subunit and suppression of binding of tRNA and mRNA-ribosome complex	Activity of ribosome protection proteins (otrA and tetM) Activity of efflux pumps (Tet, Otr, and Tap)	Most species of NTM	Most species of NTM
	Tigecycline	Binding to 30S ribosomal subunit and suppression of acyltRNA binding	Tet(X) enzyme	*M. abscessus* *M. chelonae*	Not determined for NTM species
	Rifampin	Suppression of DNA-dependent RNA polymerase of bacteria	Mutation in *rpoB* Expression of *arr*	MAC *M. kansasii*	MAC *M. kansasii* *M. ulcerans* *M. smegmatis* *M. abscessus*

Suppression of respiratory chain	Bedaquiline	Suppression of *atpE* gene, a mycobacterial ATP synthase, and lack of ATP production	Mutations in *atpE*, *mmpT5*, and *pepQ*	MDR-TB MAC *M. leprae* *M. avium* *M. abscessus* *M. massiliense*	*M. avium* *M. kansasii* *M. abscessus* *M. fortuitum* *M. flavescens* *M. massiliense* *M. intracellulare*
	Clofazimine	Suppression of bacterial proliferation by blocking the intracellular redox cycling	Mutation in *mmpR5* and *pepQ*	Most species of NTM	*M. tuberculosis* *M. abscessus* *M. intracellulare*

^1^ *M. avium* complex; ^2^penicillin-binding proteins; ^3^multidrug-resistant tuberculosis.

## Data Availability

No data were used to support this study.

## References

[1] Abubakar I., Gupta R. K., Rangaka M. X., Lipman M. (2018). Update in tuberculosis and nontuberculous mycobacteria.

[2] Nour-Neamatollahie A., Ebrahimzadeh N., Siadat S. D. (2017). Distribution of non-tuberculosis mycobacteria strains from suspected tuberculosis patients by heat shock protein 65 PCR-RFLP. *Saudi journal of biological sciences*.

[3] Sakhaee F., Vaziri F., Bahramali G., Taremian K., Siadat S. D., Fateh A. (2019). Pulmonary infection associated with Mycobacterium canariasensein suspected tuberculosis patient, Iran. *Emerging Infectious Diseases*.

[4] Smirnova T., Ustinova V., Andreevskaya S. (2021). Evaluation of a new assay for nontuberculous mycobacteria species identification in diagnostic material and cultures. *Tuberculosis*.

[5] Ratnatunga C. N., Lutzky V. P., Kupz A. (2020). The rise of non-tuberculosis mycobacterial lung disease. *Frontiers in Immunology*.

[6] Mortazavi Z., Bahrmand A., Sakhaee F. (2019). Evaluating the clinical significance of nontuberculous mycobacteria isolated from respiratory samples in Iran: an often overlooked disease. *Infection and drug resistance*.

[7] Huang W.-C., Yu M.-C., Huang Y.-W. (2020). Identification and drug susceptibility testing for nontuberculous mycobacteria. *Journal of the Formosan Medical Association*.

[8] Haworth C. S., Banks J., Capstick T. (2017). British Thoracic Society guidelines for the management of non-tuberculous mycobacterial pulmonary disease (NTM-PD). *Thorax*.

[9] Davari M., Irandoost M., Sakhaee F. (2019). Genetic diversity and prevalence of nontuberculous mycobacteria isolated from clinical samples in Tehran, Iran. *Microbial Drug Resistance*.

[10] Huh H. J., Kim S. Y., Jhun B. W., Shin S. J., Koh W. J. (2019). Recent advances in molecular diagnostics and understanding mechanisms of drug resistance in nontuberculous mycobacterial diseases. *Infection, Genetics and Evolution*.

[11] Chalmers J., Aksamit T., Carvalho A. C. C., Rendon A., Franco I. (2018). Non-tuberculous mycobacterial pulmonary infections. *Pulmonology*.

[12] Brill F., Lenz J., Lach C. (2021). Improved method for tuberculocidal and mycobactericidal activity testing of disinfectants based on the European Standard EN 14348. *Journal of Hospital Infection*.

[13] van Ingen J. (2019). Drug susceptibility testing of nontuberculous mycobacteria. *Nontuberculous Mycobacterial Disease*.

[14] Koh W. J. (2017). Nontuberculous mycobacteria-overview. *Microbiology Spectrum*.

[15] Wu M.-L., Aziz D. B., Dartois V., Dick T. (2018). NTM drug discovery: status, gaps and the way forward.. *Drug Discovery Today*.

[16] Shetye G. S., Franzblau S. G., Cho S. (2020). New tuberculosis drug targets, their inhibitors, and potential therapeutic impact. *Translational Research*.

[17] Griffith D. E., Aksamit T., Brown-Elliott B. A. (2007). An official ATS/IDSA statement: diagnosis, treatment, and prevention of nontuberculous mycobacterial diseases. *American Journal of Respiratory and Critical Care Medicine*.

[18] Floto R. A., Olivier K. N., Saiman L. (2016). US Cystic Fibrosis Foundation and European Cystic Fibrosis Society consensus recommendations for the management of non-tuberculous mycobacteria in individuals with cystic fibrosis. *Thorax*.

[19] Jarand J., Levin A., Zhang L., Huitt G., Mitchell J. D., Daley C. L. (2011). Clinical and microbiologic outcomes in patients receiving treatment for Mycobacterium abscessus pulmonary disease. *Clinical Infectious Diseases*.

[20] Brown-Elliott B. A., Nash K. A., Wallace R. J. (2012). Antimicrobial susceptibility testing, drug resistance mechanisms, and therapy of infections with nontuberculous mycobacteria. *Clinical Microbiology Reviews*.

[21] Lu M., Fitzgerald D., Karpelowsky J. (2018). Surgery in nontuberculous mycobacteria pulmonary disease. *Breathe*.

[22] Sun Q., Xiao T. Y., Liu H. C. (2018). Mutations within embCAB are associated with variable level of ethambutol resistance in Mycobacterium tuberculosis isolates from China. *Breathe*.

[23] Bakuła Z., Modrzejewska M., Pennings L. (2018). Drug susceptibility profiling and genetic determinants of drug resistance in Mycobacterium kansasii. *Antimicrobial Agents and Chemotherapy*.

[24] Xiang X., Gong Z., Deng W., Sun Q., Xie J. (2021). Mycobacterial ethambutol responsive genes and implications in antibiotics resistance. *Journal of Drug Targeting*.

[25] Fattorini L., Orefici G., Jin S. H. (1992). Resistance to beta-lactams in Mycobacterium fortuitum. *Antimicrobial Agents and Chemotherapy*.

[26] Jarlier V., Gutmann L., Nikaido H. (1991). Interplay of cell wall barrier and beta-lactamase activity determines high resistance to beta-lactam antibiotics in Mycobacterium chelonae. *Antimicrobial Agents and Chemotherapy*.

[27] Mukhopadhyay S., Chakrabarti P. (1997). Altered permeability and beta-lactam resistance in a mutant of Mycobacterium smegmatis. *Antimicrobial Agents and Chemotherapy*.

[28] Lavollay M., Fourgeaud M., Herrmann J. L. (2011). The peptidoglycan of Mycobacterium abscessus is predominantly cross-linked byl,d-transpeptidases. *Journal of Bacteriology*.

[29] Story-Roller E., Maggioncalda E. C., Cohen K. A., Lamichhane G. (2018). Mycobacterium abscessus and *β*-lactams: emerging insights and potential opportunities. *Frontiers in Microbiology*.

[30] Haworth C. S., Banks J., Capstick T. (2017). British Thoracic Society guideline for the management of non-tuberculous mycobacterial pulmonary disease (NTM-PD). *BMJ Open Respiratory Research*.

[31] Cantelli C. R., Dassonville-Klimpt A., Sonnet P. (2021). A review of current and promising nontuberculous mycobacteria antibiotics. *Future Medicinal Chemistry*.

[32] Wiseman B., Carpena X., Feliz M. (2010). Isonicotinic acid hydrazide conversion to isonicotinyl-NAD by catalase-peroxidases. *Journal of Biological Chemistry*.

[33] Rindi L. (2020). Efflux pump inhibitors against nontuberculous mycobacteria. *International Journal of Molecular Sciences*.

[34] Danilchanka O., Pavlenok M., Niederweis M. (2008). Role of porins for uptake of antibiotics by Mycobacterium smegmatis. *Antimicrobial Agents and Chemotherapy*.

[35] Heidary M., Khoshnood S., Taki E. (2021). Mechanism of action, resistance, synergism, and clinical implications of delamanid against multi drug-resistant Mycobacterium tuberculosis. *Frontiers in Microbiology*.

[36] Krieger D., Schönfeld N., Vesenbeckh S. (2016). Is delamanid a potential agent in the treatment of diseases caused by Mycobacterium avium-intracellulare?. *European Respiratory Journal*.

[37] Kim D. H., Jhun B. W., Moon S. M. (2019). In vitro activity of bedaquiline and delamanid against nontuberculous mycobacteria, including macrolide-resistant clinical isolates. *Antimicrobial Agents and Chemotherapy*.

[38] Yu X., Gao X. P., Li C. (2019). In vitro activities of bedaquiline and delamanid against nontuberculous mycobacteria isolated in Beijing, China. *Antimicrobial Agents and Chemotherapy*.

[39] Coll F., Phelan J., Hill-Cawthorne G. A. (2018). Genome-wide analysis of multi-and extensively drug-resistant Mycobacterium tuberculosis. *Nature Genetics*.

[40] Kim S.-Y., Jhun B. W., Moon S. M. (2018). Mutations ingyrA and gyrB in moxifloxacin-resistant Mycobacterium avium complex and Mycobacterium abscessus complex clinical isolates. *Antimicrobial Agents and Chemotherapy*.

[41] Lee S. H., Yoo H. K., Kim S. H. (2014). The drug resistance profile of Mycobacterium abscessus group strains from Korea. *Annals of Laboratory Medicine*.

[42] Esteban J., Martín-de-Hijas N. Z., Ortiz A. (2009). Detection of lfrA and tap efflux pump genes among clinical isolates of non-pigmented rapidly growing mycobacteria. *International Journal of Antimicrobial Agents*.

[43] Sköld O. E., Swedberg G. (2017). Sulfonamides and trimethoprim. Antimicrobial drug resistance. *Sulfonamides and trimethoprim*.

[44] Sirawaraporn W., Sirawaraporn R., Chanpongsri A., Jacobs W. R., Santi D. V. (1991). Purification and characterization of dihydrofolate reductase from wild-type and trimethoprim-resistant Mycobacterium smegmatis. *Experimental Parasitology*.

[45] Shoen C., DeStefano M., Pucci M., Cynamon M. H. Evaluating the sterilizing activity of SPR720 in combination therapy against Mycobacterium tuberculosis infection in mice.

[46] Locher C. P., Jones S. M., Hanzelka B. L. (2015). A novel inhibitor of gyrase B is a potent drug candidate for treatment of tuberculosis and nontuberculosis mycobacterial infections. *Antimicrobial Agents and Chemotherapy*.

[47] Brown-Elliott B. A., Rubio A., Wallace R. J. (2018). Antimicrobial Agents and Chemotherapy.

[48] Hirama T., Shiono A., Egashira H. (2016). PCR-based rapid identification system using bridged nucleic acids for detection of clarithromycin-resistant Mycobacterium avium-M. intracellulare complex isolates. *Journal of Clinical Microbiology*.

[49] Jhaveri V. V., Singhal D., Riedel S., Rowley C. F., Nathavitharana R. R. (2020). Surgical cure of clarithromycin resistant _Mycobacterium chelonae_ breast implant infection: a case report and review of the literature. *Journal of Clinical Tuberculosis and Other Mycobacterial Diseases*.

[50] Bastian S., Veziris N., Roux A. L. (2011). Assessment of clarithromycin susceptibility in strains belonging to the Mycobacterium abscessus group by erm (41) and rrl sequencing. *Antimicrobial Agents and Chemotherapy*.

[51] Nash K. A., Brown-Elliott B. A., Wallace R. J. (2009). A novel gene, erm(41), confers inducible macrolide resistance to clinical isolates of Mycobacterium abscessus but is absent from Mycobacterium chelonae. *Antimicrobial Agents and Chemotherapy*.

[52] Kim S. Y., Kim C. K., Bae I. K. (2015). The drug susceptibility profile and inducible resistance to macrolides of Mycobacterium abscessus and Mycobacterium massiliense in Korea. *Diagnostic Microbiology and Infectious Disease*.

[53] Koh W.-J., Jeong B. H., Jeon K. (2016). Oral macrolide therapy following short-term combination antibiotic treatment of Mycobacterium massiliense lung disease. *Chest*.

[54] Shallom S. J., Moura N. S., Olivier K. N., Sampaio E. P., Holland S. M., Zelazny A. M. (2015). New real-time PCR assays for detection of inducible and acquired clarithromycin resistance in the Mycobacterium abscessus group. *Journal of Clinical Microbiology*.

[55] Winthrop K. L., Ku J. H., Marras T. K. (2015). The tolerability of linezolid in the treatment of nontuberculous mycobacterial disease. *European Respiratory Journal*.

[56] McNeil M. B., Dennison D. D., Shelton C. D., Parish T. (2017). In vitro isolation and characterization of oxazolidinone-resistant Mycobacterium tuberculosis. *Antimicrobial Agents and Chemotherapy*.

[57] Yuste J. R., Bertó J., Del Pozo J. L., Leiva J. (2017). Prolonged use of tedizolid in a pulmonary non-tuberculous mycobacterial infection after linezolid-induced toxicity.. *Journal of Antimicrobial Chemotherapy*.

[58] Kim T. S., Choe J. H., Kim Y. J. (2017). Activity of LCB01-0371, a novel oxazolidinone, against Mycobacterium abscessus. *Antimicrobial Agents and Chemotherapy*.

[59] Yagi K., Ishii M., Namkoong H. (2017). The efficacy, safety, and feasibility of inhaled amikacin for the treatment of difficult-to-treat non-tuberculous mycobacterial lung diseases. *BMC Infectious Diseases*.

[60] Brown-Elliott B. A., Iakhiaeva E., Griffith D. E. (2013). In vitro activity of amikacin against isolates of Mycobacterium avium complex with proposed MIC breakpoints and finding of a 16S rRNA gene mutation in treated isolates. *Journal of Clinical Microbiology*.

[61] Nessar R., Reyrat J. M., Murray A., Gicquel B. (2011). Genetic analysis of new 16S rRNA mutations conferring aminoglycoside resistance in Mycobacterium abscessus. *Journal of Antimicrobial Chemotherapy*.

[62] Raaijmakers J., Schildkraut J. A., Hoefsloot W., van Ingen J. (2021). The role of amikacin in the treatment of nontuberculous mycobacterial disease. *Expert Opinion on Pharmacotherapy*.

[63] Brodersen D. E., Clemons W. M., Carter A. P., Morgan-Warren R. J., Wimberly B. T., Ramakrishnan V. (2000). The structural basis for the action of the antibiotics tetracycline, pactamycin, and hygromycin B on the 30S ribosomal subunit. *Cell*.

[64] Roberts M. C. (2005). Update on acquired tetracycline resistance genes. *FEMS Microbiology Letters*.

[65] Ramón-García S., Martín C., Aínsa J. A., de Rossi E. (2006). Characterization of tetracycline resistance mediated by the efflux pump Tap from Mycobacterium fortuitum. *Journal of Antimicrobial Chemotherapy*.

[66] Wallace R. J., Dukart G., Brown-Elliott B. A., Griffith D. E., Scerpella E. G., Marshall B. (2014). Clinical experience in 52 patients with tigecycline-containing regimens for salvage treatment of Mycobacterium abscessus and Mycobacterium chelonae infections. *Journal of Antimicrobial Chemotherapy*.

[67] Cui C.-Y., He Q., Jia Q. L. (2021). Evolutionary trajectory of the Tet (X) family: critical residue changes towards high-level tigecycline resistance. *Msystems*.

[68] Miotto P., Tessema B., Tagliani E. (2017). A standardised method for interpreting the association between mutations and phenotypic drug resistance in Mycobacterium tuberculosis. *European Respiratory Journal*.

[69] Yoshida S., Suzuki K., Tsuyuguchi K. (2006). Detection of rpoB mutations in rifampicin-resistant Mycobacterium kansasii. *Kekkaku (Tuberculosis)*.

[70] Philley J. V., Wallace R. J., Benwill J. L. (2015). Preliminary results of bedaquiline as salvage therapy for patients with nontuberculous mycobacterial lung disease. *Chest*.

[71] Pang Y., Zheng H., Tan Y., Song Y., Zhao Y. (2017). In vitro activity of bedaquiline against nontuberculous mycobacteria in China. *Antimicrobial Agents and Chemotherapy*.

[72] Deoghare S. (2013). Bedaquiline: a new drug approved for treatment of multidrug-resistant tuberculosis. *Indian Journal of Pharmacology*.

[73] Koul A., Dendouga N., Vergauwen K. (2007). Diarylquinolines target subunit c of mycobacterial ATP synthase. *Nature Chemical Biology*.

[74] Alexander D. C., Vasireddy R., Vasireddy S. (2017). Emergence of mmpT5 variants during bedaquiline treatment of Mycobacterium intracellulare lung disease. *Journal of Clinical Microbiology*.

[75] Aguilar-Ayala D. A., Cnockaert M., André E. (2017). Journal of Medical Microbiology.

[76] Almeida D., Ioerger T., Tyagi S. (2016). Mutations in pepQ confer low-level resistance to bedaquiline and clofazimine in Mycobacterium tuberculosis. *Antimicrobial Agents and Chemotherapy*.

[77] Martiniano S. L., Wagner B. D., Levin A., Nick J. A., Sagel S. D., Daley C. L. (2017). Safety and effectiveness of clofazimine for primary and refractory nontuberculous mycobacterial infection. *Chest*.

[78] Pfaeffle H. O., Alameer R. M., Marshall M. H., Houpt E. R., Albon D. P., Heysell S. K. (2021). Clofazimine for treatment of multidrug-resistant non-tuberculous mycobacteria. *Pulmonary Pharmacology & Therapeutics*.

[79] Zhang S., Chen J., Cui P., Shi W., Zhang W., Zhang Y. (2015). Identification of novel mutations associated with clofazimine resistance in Mycobacterium tuberculosis. *Journal of Antimicrobial Chemotherapy*.

[80] Chen Y., Chen J., Zhang S. (2018). Novel mutations associated with clofazimine resistance in Mycobacterium abscessus. *Antimicrobial Agents and Chemotherapy*.

[81] Luo J., Yu X., Jiang G. (2018). In vitro activity of clofazimine against nontuberculous mycobacteria isolated in Beijing, China. *Antimicrobial Agents and Chemotherapy*.

[82] Falkinham J. O. (2015). Environmental sources of nontuberculous mycobacteria. *Clinics in Chest Medicine*.

[83] Edirisinghe E. R., Dissanayake D. A., Abayasekera C. L., Arulkanthan A. (2017). Efficacy of calcium hypochlorite and ultraviolet irradiation against Mycobacterium fortuitum and Mycobacterium marinum. *Mycobacteriology*.

[84] Aranke M., Moheimani R., Phuphanich M. (2021). Disinfectants in interventional practices. *Current Pain and Headache Reports*.

[85] Paliy A., Zavgorodnii A. I., Kalashnyk M. V. (2020). Influence of new frost-resistant disinfectant on the ultrastructural organization of atypical mycobacteria. Ukrainian. *Journal of Ecology*.

[86] Bohrerova Z., Linden K. G. (2006). Ultraviolet and chlorine disinfection of Mycobacterium in wastewater: effect of aggregation. *Water Environment Research*.

[87] Wang J., Sui M., Yuan B., Li H., Lu H. (2019). Inactivation of two Mycobacteria by free chlorine: effectiveness, influencing factors, and mechanisms. *Science of the Total Environment*.

[88] Lee E. S., Lee M. H., Kim B. S. (2015). Evaluation of propidium monoazide-quantitative PCR to detect viable _Mycobacterium fortuitum_ after chlorine, ozone, and ultraviolet disinfection. *International Journal of Food Microbiology*.

[89] Chen Y. Q., Chao C. H. E. N., Zhang X. J., Zheng Q., Liu Y. Y. (2012). Inactivation of resistant Mycobacteria mucogenicum in water: chlorine resistance and mechanism analysis. *Biomedical and Environmental Sciences*.

[90] Steber J., Schröder F. R. (1997). Glucoprotamin [R]-an antimicrobial agent with favourable biodegradation properties. *Hygiene Und Medizin*.

[91] Holton J., Nye P., McDonald V. (1994). Efficacy of selected disinfectants against Mycobacteria and Cryptosporidia. *Journal of Hospital Infection*.

[92] Cortesia C., Vilchèze C., Bernut A. (2014). Acetic acid, the active component of vinegar, is an effective tuberculocidal disinfectant. *MBio*.

[93] David H. L., Jones W. D., Newman C. M. (1971). Ultraviolet light inactivation and photoreactivation in the mycobacteria. *Infection and Immunity*.

[94] Lee E.-S., Yoon T. H., Lee M. Y., Han S. H., Ka J. O. (2010). Inactivation of environmental mycobacteria by free chlorine and UV. *Water Research*.

[95] Hayes S., Sivaganesan M., White K. M., Pfaller S. L. (2008). Assessing the effectiveness of low-pressure ultraviolet light for inactivating Mycobacterium avium complex (MAC) micro-organisms. *Letters in Applied Microbiology*.

[96] Jacobs J. M., Lazur A., Baya A. (2004). Publication number UM-SG-SGEP, Finfish Worksheet, Prevention and disinfection of Mycobacterium sp. in aquaculture. *Maryland Sea Grant Extension Publication*.

[97] de Carvalho C. C., Teixeira R., Fernandes P. (2020). Mycobacterium vaccae adaptation to disinfectants and hand sanitisers, and evaluation of cross-tolerance with antimicrobials. *Antibiotics*.

[98] Selvaraju S. B., Khan I. U., Yadav J. S. (2005). Biocidal activity of formaldehyde and nonformaldehyde biocides toward Mycobacterium immunogenum and Pseudomonas fluorescens in pure and mixed suspensions in synthetic metalworking fluid and saline. *Applied and Environmental Microbiology*.

[99] van Ingen J. (2015). Microbiological diagnosis of nontuberculous mycobacterial pulmonary disease. *Clinics in Chest Medicine*.

[100] Canetti G., Froman S., Grosset J. A. (1963). Mycobacteria: laboratory methods for testing drug sensitivity and resistance. *Bulletin of the World Health Organization*.

[101] Research Committee of the British Thoracic Society (2001). First randomised trial of treatments for pulmonary disease caused by M avium intracellulare, M malmoense, and M xenopi in HIV negative patients: rifampicin, ethambutol and isoniazid versus rifampicin and ethambutol.

[102] Van Ingen J., van der Laan T., Dekhuijzen R., Boeree M., van Soolingen D. (2010). In vitro drug susceptibility of 2275 clinical non-tuberculous Mycobacterium isolates of 49 species in The Netherlands. *International Journal of Antimicrobial Agents*.

[103] Wallace R., Nash D. R., Steele L. C., Steingrube V. (1986). Susceptibility testing of slowly growing mycobacteria by a microdilution MIC method with 7H9 broth. *Journal of Clinical Microbiology*.

[104] van Ingen J., Boeree M. J., van Soolingen D., Mouton J. W. (2012). Resistance mechanisms and drug susceptibility testing of nontuberculous mycobacteria. *Drug Resistance Updates*.

[105] Stone M., Wallace R. J., Swenson J. M., Thornsberry C., Christensen L. A. (1983). Agar disk elution method for susceptibility testing of Mycobacterium marinum and Mycobacterium fortuitum complex to sulfonamides and antibiotics. *Antimicrobial Agents and Chemotherapy*.

